The article "Curcumin alleviates acute kidney injury in a dry‐heat environment by reducing oxidative stress and inflammation in a rat model" was published in 2020. Journal: J Biochem Mol Toxicol.

# Curcumin alleviates acute kidney injury in a dry‐heat environment by reducing oxidative stress and inflammation in a rat model

**DOI:** 10.1002/jbt.22630

**Published:** 2020-09-12

**Authors:** Yin‐Hui Zhao, Cai‐Fu Shen, Guang‐Jun Wang, Yan Kang, Yun‐Hong Song, Jiang‐Wei Liu

**Affiliations:** ^1^ Key Laboratory of the Special Environmental Medicine of Xinjiang General Hospital of Xinjiang Military of the PLA Urumuqi China; ^2^ Emergency Critical Department Shanghai General Hospital Shanghai China; ^3^ Department of Ultrasound 69240 Army Hospital of PLA Urumqi Xinjiang China

**Keywords:** acute renal injury, curcumin, dry‐heat environment, inflammatory reaction, oxidative stress

## Abstract

Curcumin exhibits anti‐inflammatory and antioxidant activities. We investigated the protective effects of curcumin in a renal injury rat model under dry‐heat conditions. We divided Sprague‐Dawley rats into four groups: dry‐heat 0‐ (normal temperature control group), 50‐, 100‐, and 150‐minute groups. Each group was divided into five subgroups (n = 10): normal saline (NS), sodium carboxymethylcellulose (CMCNa), and curcumin pretreated low, medium, and high‐dose (50, 100, and 200 mg/kg, respectively) groups. Compared to the normal temperature group, serum creatinine, blood urea nitrogen, urinary kidney injury molecule‐1, and neutrophil gelatinase‐associated load changes in lipoprotein (NGAL) levels were significantly increased in the dry‐heat environment group (*P* < .05); inducible nitric oxide synthase (iNOS) and cyclooxygenase‐2 (COX‐2) expression and malondialdehyde (MDA) and related inflammatory factor levels were increased in the kidney tissue. Superoxide dismutase (SOD) and catalase (CAT) levels were decreased. However, following all curcumin pretreatment, the serum levels of kidney injury indicators and NGAL were decreased in the urine compared to those in the NS and CMCNa groups (*P* < .05), whereas renal SOD and CAT activities were increased and MDA was decreased (*P* < .05). Renal tissues of the 150‐minute group showed obvious pathological changes. Compared to the NS group, pathological changes in the renal tissues of the 100‐ and 200‐mg/kg curcumin groups were significantly reduced. Furthermore, iNOS and COX‐2 expression and inflammatory factor levels were decreased after curcumin treatment. Curcumin exerted renoprotective effects that were likely mediated by its antioxidant and anti‐inflammatory effects in a dry‐heat environment rat model.

## 1 INTRODUCTION

Heatstroke is a fatal disease characterized by disorders of the central nervous system^[^ ^1^, ^2^ ^]^ such as delirium and convulsions and a core body temperature ≥40℃. As early as 2002, a new definition was proposed for heatstroke, describing the condition as multiple organ dysfunction caused by thermal cell toxicity, systemic inflammatory response syndrome, and coagulation disorders.^[^ ^3^ ^]^ Heatstroke often occurs under high‐temperature conditions, particularly in dry‐heat desert environments with high temperatures, low humidity, and strong ultraviolet radiation. In special workers, combatants, and travelers in the desert, heatstroke is often accompanied by severe fluid loss and other serious consequences.

Acute kidney injury (AKI) is a common complication of heatstroke. AKI presents as the sudden onset of renal parenchymal injury,^[^ ^4^ ^]^ and the pathogenesis of heatstroke‐associated AKI likely involves decreased perfusion caused by dehydration and hypovolemia, direct thermal injury, rhabdomyolysis‐associated myoglobinuria, and systemic inflammatory response syndrome.^[^ ^5^ ^]^ In addition, previous studies showed that the concentrations of circulating inflammatory cytokines including interleukin (IL)‐6, tumor necrosis factor (TNF)‐α, and IL‐1β were markedly increased and histological examination showed widespread hemorrhage, thrombosis, and migration of leukocytes in both animals and patients with severe heatstroke.^[^ ^6^, ^7^, ^8^ ^]^ Inducible nitric oxide synthase (iNOS) and cyclooxygenase (COX)‐2 are the primary factors that cause inflammation and oxidative stress.

Curcumin is a widely used dietary pigment and, according to previous studies, exerts pharmacological effects such as anti‐inflammation and antioxidation.^[^ ^9^ ^]^ Abdel‐Moneim et al^[^ ^10^ ^]^ found that curcumin significantly reduced the activity of malondialdehyde (MDA) in the renal tissue of rats with acute renal injury induced by Pb^2+^, which is involved in antioxidative stress. Hismiogullari^[^ ^11^ ^]^ and Kim et al^[^ ^12^ ^]^ also found that curcumin reduced the activity of MDA and improved superoxide dismutase (SOD) and catalase (CAT) activities in acute/chronic renal injury in experimental animals. Studies have shown that curcumin can reduce the expression of iNOS and COX‐2 to inhibit inflammatory reactions.^[^ ^13^ ^]^ However, few studies have focused on the renal protective effects of curcumin in a dry‐heat environment. Therefore, in this study, we predicted that curcumin exerts protective effects on the kidney by suppressing oxidative stress and inflammation and that pretreated groups would show improved heat resistance and protection against organ injury. We examined the renoprotective effects of curcumin in a rat model of the dry‐heat environment and possible underlying mechanisms of action.

## 2 MATERIALS AND METHODS

### 2.1 Animals

A total of 200 male Sprague‐Dawley (SD) rats (65‐70 days old, weighing 190‐220 g) were purchased from the Experimental Animal Center of Xinjiang Medical University. Animals were housed individually at 22℃ with 35% humidity on a 12‐hour light/dark cycle. The rats were fed a standard pellet diet and provided water ad libitum. This study was approved by the ethical committee of the General Hospital of the Xinjiang Military Region of the PLA. Animal care and experiments were conducted according to the National Science Council guidelines.

### 2.2 Establishment of the heatstroke rat model, pretreatment, and collection of blood, urine, and kidney tissue

The 200 SD rats were randomly divided into four groups (n = 50): dry‐heat 0‐ (normal temperature control), 50‐, 100‐, and 150‐minute groups. Each time point group was further divided into five subgroups (n = 10): normal saline (NS); sodium carboxymethylcellulose (CMCNa); and curcumin‐treated low‐, medium, and high‐dose (50, 100, and 200 mg/kg, respectively) groups. The NS, CMCNa, and curcumin‐treated groups rats were administered 0.9% saline, 0.5% CMCNa solution, and graded oral doses of curcumin in 0.5% CMCNa solution, respectively, by gavage once daily for 7 consecutive days.

The heat‐dry heatstroke rat model was established as reported previously for a heatstroke model in a desert dry‐heat environment.^[^ ^14^ ^]^ Rats in the normal temperature control group were placed at room temperature (20℃ ± 2℃) with humidity at 40% to 50%. The remaining rats were placed in a dry‐heat environment (simulated climate cabin for the special environment of Northwest China, Urumqi, China) at 41℃ ± 0.5℃ and humidity of 10% ± 1%. The core body temperature of the rats was monitored every 30 minutes and the rats were removed from the experimental cabin at 50, 100, and 150 minutes according to the grouping. The rats were then anesthetized with 3% pentobarbital sodium and killed, after which blood was collected from the inferior vena cava to analyze blood indices, urine was collected for renal damage index analysis by puncturing the bladder, and the renal tissue was stored at −80℃ until analysis.

### 2.3 Determination of serum creatinine and urea in rats

The serum was separated by centrifuging the blood samples for 10 minutes at 1500*g*, and *was* stored at −20°C until analyses of creatinine (Cr) and blood urea nitrogen (BUN) levels with an automatic biochemical analyzer (BS‐180; Shenzhen Mindray Bio‐Medical Electronics Co, Ltd, Shenzhen, China).

### 2.4 Preparation of kidney tissue homogenate

Kidney tissue samples (0.1 ± 0.05 g) were placed in a glass homogenizer and cut into small pieces using sharp scissors. Next, 200 µL phosphate‐buffered solution was added and the kidney tissue was finely ground, followed by addition of 700‐µL phosphate‐buffered solution to obtain a homogenate concentration of 10%. The homogenate was stored at −20℃ until analysis of MDA. The homogenate was separated by centrifugation for 10 min at 1500*g*; the supernatant was collected and stored at −20℃ for further analysis of SOD, CAT, and inflammatory factors. The whole procedure was performed on ice.

### 2.5 Determination of total protein in renal homogenate by BCA

The renal tissue homogenate was diluted from 10% to 0.5% with phosphate‐buffered saline and mixed well. The working fluid was prepared according to the instructions (A solution:B solution = 50:1), mixed well, and stored at 4°C for 24 hours (kits were provided by Thermo Fisher Scientific, Waltham, MA). Protein standards and samples of different concentrations were then added to 96‐well plates. The working solution (200 µL) was added to each well, and the plate was sealed and placed in a water bath at 37°C for 30 minutes. The data were recorded, a standard curve was drawn, and protein content was calculated.

### 2.6 Determination of SOD and CAT activity and MDA levels in kidney tissue

The SOD and CAT activity and MDA levels in the kidney tissue were measured with commercial kits (Nanjing Jiancheng Bioengineering Institute, Nanjing, China). SOD and CAT were measured using the xanthine oxidase method and visible spectrometry (OD_405_ and OD_510_ nm), respectively, and the results were expressed in units per microgram. MDA was measured using the thiobarbituric acid method and the results were expressed in millimole per milligram protein.

### 2.7 Measurement of urinary kidney injury molecule‐1 and neutrophil gelatinase‐associated load changes in lipoprotein and inflammatory factors in kidney tissue

The urinary contents of kidney injury molecule‐1 (KIM‐1) and neutrophil gelatinase‐associated load changes in lipoprotein (NGAL) were measured using commercial Enzyme‐Linked Immunosorbent Assay (ELISA) Kits (Anhui Qiaoyi Biotechnology, Anhui, China). IL‐1β, IL‐6, and TNF‐α levels in the kidney tissue were measured using commercial ELISA Kits (Anhui Qiaoyi Biotechnology) according to the manufacturer's instructions.

### 2.8 Western blot analysis

The kidney samples were ground with liquid nitrogen and lysed with lysis buffer for 2 hours on ice. The extract was centrifuged for 20 minutes at 2500*g*, the supernatant was collected and stored in Eppendorf tubes at −80℃. The samples were mixed with 2X loading buffer and boiled for 8 minutes before separation by electrophoresis. The amounts of protein were measured using the bicinchoninic method. The amount of protein loaded for electrophoresis was 120 ng. Separation was performed at a voltage of 60 V, followed by 100 V for 1.5 hours and electrotransfer to a polyvinylidene fluoride membrane for 20 to 30 minutes according to different molecular weights. The membrane was blocked with 5% nonfat milk powder for 2 hours at room temperature and then incubated with the primary antibody overnight at 4℃, followed by the secondary antibody for 1 hour at room temperature. The target band was detected by chemiluminescence, and the protein was semiquantified by analyzing the gray intensity.

### 2.9 Histopathological examination

The kidney tissue samples were fixed in 10% neutral‐buffered formalin, dehydrated with graded alcohol concentrations, cleared with xylene, embedded in paraffin, and cut into 5‐µm‐thick sections, which were stained with hematoxylin and eosin. After mounting on slides, the sections were reviewed blindly and scored using Paller's score.^[^ ^15^ ^]^ Samples from each rat were randomly selected, and 10 visual fields were analyzed at ×400 magnification under a light microscope; 100 visual fields were selected from each group. The scoring criteria were the presence and extent of tubular epithelial cell flattening (one point), brush border loss (one point), cell membrane bleb formation (one or two points), interstitial edema (one point), cytoplasmic vacuolization (one point), cell necrosis (one or two points), and tubular lumen obstruction (one or two points).

### 2.10 Statistical analysis

Because we performed repeated measurements, repeated measurement analysis of variance was used to compare differences between groups and time points. Intergroup and intragroup data were analyzed by one‐way analysis of variance after performing the necessary transformation of data that were not normally distributed (SPSS, version 21.0; SPSS, Inc, Chicago, IL). The effect was considered significant at a *P* < .05.

## 3 RESULTS

### 3.1 Cr, BUN, KIM‐1, and NGAL analysis

Figure 1 shows that the plasma Cr and BUN levels were significantly increased in rats exposed to a dry‐heat environment compared to those in the normal temperature group for a prolonged time. Pretreatment with different doses of curcumin prevented the increase in BUN and Cr compared to in the NS and CMCNa groups (*P* < .05; Figure 1A,B). Indicators of early renal injury, KIM‐1 and NGAL in the urine, showed the same trend as Cr and BUN (*P* < .05; Figure 1C,D).

**Figure 1:** Effect of curcumin on renal injury indicators in heatstroke rat model alterations. Values represent the mean ± standard error of 10 rats, analyzed by one‐way analysis of variance. *P < .05 compared to normal saline (NS) control groups at the same time point. ^#^ *P* < .05 compared to the 0‐minute groups among the NS control groups. BUN, blood urea nitrogen; KIM‐1, kidney injury molecule‐1; NGAL, neutrophil gelatinase‐associated load changes in lipoprotein

### 3.2 SOD and CAT activities and MDA levels in the kidney tissue

Figure 2 shows that increasing the degree of heatstroke significantly (*P* < .05) decreased SOD and CAT activities (Figure 2A,B); MDA levels were increased in the kidney tissue (Figure 1C) in the NS and CMCNa groups. Treatment with different doses of curcumin at a normal temperature did not significantly change the SOD and CAT activities or MDA levels compared to those in the NS and CMCNa groups. Significant recovery of SOD and CAT and suppression of MDA levels were observed in response to treatment with different doses of curcumin in the dry‐heat environment.

**Figure 2:** Effect of curcumin on renal enzyme activities in heatstroke rat model alterations. Values represent the mean ± standard error of 10 rats, analyzed by one‐way analysis of variance. *P < .05 compared to normal saline (NS) groups at the same time points. ^#^ *P* < .05 compared to the 0‐minute groups among the NS control groups. CAT, catalase; MDA, malondialdehyde; SOD, superoxide dismutase

### 3.3 Contents of inflammatory factors in the kidney tissue

Inflammatory factors were also detected in the rat model of heatstroke (Figure 3). We observed decreased levels of IL‐6, IL‐1β, and TNF‐α in groups pretreated with different doses of curcumin compared to those in the NS and CMCNa groups (*P* < .05). Inflammatory factor levels increased with increasing levels and periods of heatstroke (*P* < .05). Notably, inflammatory factor levels decreased significantly in curcumin pretreated groups at 150 minutes compared to those in the NS group.

**Figure 3:** Effect of curcumin on renal inflammatory factors in heatstroke rat model alterations. Values represent the mean ± standard error for 10 rats, analyzed by one‐way analysis of variance. *P < .05 compared to normal saline (NS) groups. ^#^ *P* < .05 compared to the 0‐minute groups among the NS control groups. IL‐6, interleukin‐6; TNF‐α, tumor necrosis factor‐α

### 3.4 Pathological changes in kidney tissue

We selected the 150‐minute group to evaluate the protective effects of curcumin on the kidney. Figure 4 shows the pathological changes in this group. In the NS group (Figure 4A), obvious pathological changes were detected in the kidney tissue. The Bowman capsule became narrow, epithelial cells of the proximal convoluted tubules showed edema, and the lumens of the tubules became narrow. Part of the proximal convoluted tubules contained protein cast. Compared to the NS group, the curcumin 100‐ and 200‐mg/kg groups showed fewer pathological changes, particularly at 200 mg/kg at which the protein cast disappeared and epithelial cell swelling was alleviated (Figure 4B‐D). Paller's scores in the curcumin 100‐ and 200‐mg/kg groups (498.28 ± 26.33 and 386.56 ± 21.38, respectively) were significantly lower compared to that in the control group (696.45 ± 23.67; *P* < .05). The curcumin 50‐mg/kg group (696.45 ± 23.07) presented similar pathological changes as the control group, indicating that curcumin did not significantly affect the kidney (Figure 5).

**Figure 4:** Effect of curcumin on pathological changes in kidneys. A, Normal temperature group pretreated with 0.9% saline. B, Curcumin 50 mg/kg, (C) 100 mg/kg, and (D) 200 mg/kg. A‐D, magnification, ×400

**Figure 5:** Changes in Paller's score of renal tubules. Dry‐heat (DH) group at 150 minutes pretreated with 0.9% saline. *P < .05 compared to DH group

### 3.5 Expression of COX‐2 and iNOS

We chose the 150‐minute group to compare the effect of different doses of curcumin on COX‐2 and iNOS expression in the dry‐heat environment. The expression of these proteins was increased significantly in the NS group exposed to the dry‐heat environment for 150 minutes compared to the normal temperature group. The expression of COX‐2 and iNOS in the kidney tissue decreased significantly at doses of 100 and 200 mg/kg/d (*P* < .05). However, curcumin at 50 mg/kg/d did not show any difference compared to that in the NS group in the dry‐heat environment at 150 minutes (Figure 6A‐D).

**Figure 6:** Effect of curcumin on the expression of cyclooxygenase (COX)‐2 and inducible nitric oxide synthase (iNOS) in a dry‐heat environment rat model. Values represent the mean ± standard error; NT control, normal temperature group pretreated with 0.9% saline; DH control, dry‐heat group pretreated with 0.9% saline. *P < .05 and ^#^ *P* < .05 compared to NT and DH controls (*P* < .05).

## 4 DISCUSSION

Presently, there is no specific and effective treatment strategy for heatstroke. Consequently, stroke patients are often left with serious sequelae; therefore, preventing heatstroke is very important. In heatstroke, the effective circulating blood volume of the body is reduced, leading to a corresponding reduction in the blood flow to the peripheral tissues and kidney.^[^ ^16^ ^]^ Blood redistribution ensures that important organs receive blood supply. Intestinal injury causes bacteria to leak into the blood, leading to systemic inflammatory response syndrome.^[^ ^17^ ^]^ Renal ischemia and hypoxia induce oxidative stress and inflammatory reactions in the cells, and the direct cellular toxicity of heat stress further damages the kidney cells. KIM‐1 is a type 1 membrane glycoprotein highly expressed in proximal tubular cells after nephrotoxic or ischemic insults.^[^ ^18^, ^19^ ^]^ In addition, NGAL is a cytosolic protein found in the urine, blood, renal, and proximal‐distal tubules in cases of renal ischemia, presence of nephrotoxins, kidney parenchymal damage, and renal transplant denial.^[^ ^20^ ^]^ In the group not treated with curcumin, we found that KIM‐1 and NGAL levels were increased when the time of heatstroke was prolonged, confirming the presence of kidney injury related to heatstroke.

As a traditional medicine, curcumin is safe and shows few side effects. The dose of curcumin used in this study was referenced from a previous study, which explored the protective effect of curcumin on kidney injury.^[^ ^21^ ^]^ In this study, we found that the protective effect of curcumin on renal injury was mild in the 50‐mg/kg pretreatment group, and the protective effects of the 100‐ and 200‐mg/kg doses were equivalent to some indicators.

One important mechanism of heatstroke is inflammatory reactions, and most severe heatstroke patients experience multiple organ dysfunction. Curcumin has been shown to inhibit the release of numerous cytokines such as IL‐1β, IL8, TNF‐α, and IL‐6.^[^ ^22^, ^23^ ^]^ Our study revealed that curcumin reduces the release of inflammatory factors. However, the anti‐inflammatory mechanism of curcumin is not clear, and it is generally thought to be mediated by inhibition of iNOS and COX‐2 expression. In this study, curcumin pretreatment reduced iNOS and COX‐2 expression under the same conditions of heat stress in the kidney tissues, which is consistent with the results of previous studies.^[^ ^13^ ^]^

Oxidative stress is an alternate mechanism of renal damage and plays a role in the fatal pathogenesis of various diseases including myocardial ischemia, cerebral brain ischemia‐reperfusion injury, hemorrhage and shock, neuronal cell injury, hypoxia, and cancer. In this study, we compared the SOD and CAT activities and MDA levels at different periods of heatstroke without pretreatment with curcumin. We found that the MDA content increased with increasing heatstroke duration and was related to the severity of pathological changes, whereas the SOD and CAT activities showed the opposite trend. SOD and CAT are known to protect cells from oxidative stress by detoxifying carcinogens or reducing stress,^[^ ^24^ ^]^ and overproduction of reactive oxygen species alters the oxidant‐antioxidant balance. This disrupts the membrane lipid composition through lipid peroxidation and subsequently, increases MDA, a final metabolite product of lipid peroxidation.^[^ ^25^, ^26^ ^]^ In addition, curcumin has been shown to enhance CAT activity in the liver and kidney of mice.^[^ ^27^ ^]^ We found that the renal activities of CAT and SOD were enhanced in rats treated with curcumin for 7 days, suggesting an indirect antioxidant effect of curcumin. CAT and SOD activity remained unaffected by curcumin (complete treatment) in the normal temperature group, suggesting a differential effect of curcumin on the induction of renal enzymes.

Another issue of concern was that the effects of curcumin on the different indicators differed and showed dose‐dependence. In this study, we found that all indicators were significantly affected by curcumin at a dose of 200 mg/kg/d.

In summary, kidney injury induced by a dry‐heat environment in rats was characterized in this study. This is the first description of the protective effect of curcumin pretreatment against renal oxidant damage and inflammation in a dry‐heat rat model. Our data suggest that both direct and indirect antioxidant effects were involved in the observed nephroprotective effect of curcumin. The protective effect of curcumin on the kidney under the heat and dry environment in rats was defined, and we performed a preliminary study of the possible underlying mechanism. Furthermore, curcumin is insoluble in water with a low‐oral bioavailability rate; thus, we dissolved curcumin in a 0.5% CMCNa solution. The route of administration and the optimal dose of curcumin require further analysis.

## CONFLICT OF INTERESTS

The authors declare that there are no conflict of interests.
